RETRACTED

# Expression Profiling of Transcriptome and Its Associated Disease Risk in Yang Deficiency Constitution of Healthy Subjects

**DOI:** 10.1155/2016/1493098

**Published:** 2016-11-15

**Authors:** Ruoxi Yu, Yin Yang, Yuanyuan Han, Pengwei Hou, Yingshuai Li, Siqi Li, Qi Wang

**Affiliations:** ^1^Health Preservation Institute, Beijing University of Chinese Medicine, Beijing, China; ^2^Center for Studies in Constitution Research of Traditional Chinese Medicine, School of Preclinical Medicine, Beijing, China; ^3^Novel Bioinformatics Co., Ltd., Shanghai, China

## Abstract

*Objectives*. Differences among healthy subjects and associated disease risks are of substantial interest in clinical medicine. According to the theory of “constitution-disease correlation” in traditional Chinese medicine, we try to find out if there is any connection between intolerance of cold in Yang deficiency constitution and molecular evidence and if there is any gene expression basis in specific disorders.* Methods*. Peripheral blood mononuclear cells were collected from Chinese Han individuals with Yang deficiency constitution (*n* = 20) and balanced constitution (*n* = 8) (aged 18–28) and global gene expression profiles were determined between them using the Affymetrix HG-U133 Plus 2.0 array.* Results*. The results showed that when the fold change was ≥1.2 and* q* ≤ 0.05, 909 genes were upregulated in the Yang deficiency constitution, while 1189 genes were downregulated. According to our research differential genes found in Yang deficiency constitution were usually related to lower immunity, metabolic disorders, and cancer tendency.* Conclusion*. Gene expression disturbance exists in Yang deficiency constitution, which corresponds to the concept of constitution and gene classification. It also suggests people with Yang deficiency constitution are susceptible to autoimmune diseases, enteritis, arthritis, metabolism disorders, and cancer, which provides molecular evidence for the theory of “constitution-disease correlation.”

## 1. Introduction

Priority is granted to preventive medication, which is the developmental tendency of modern medicine. Traditional Chinese medicine believes that occurrence of disease depends on the quality of body constitution, which is formed in the life process based on the born gifts and acquired morphological structure. It has the integrated relatively stable peculiarity in physiological function and psychological states. The theory of constitution holds that constitution can be divided into several types. Epidemiological study in the Chinese Han population revealed nine types of constitutions: the balanced constitution and eight pathological constitutions (qi deficiency, Yang deficiency, Yin deficiency, Phlegm-dampness, damp-heat, stagnant blood, stagnant qi, and inherited special constitutions) [1].

RETRACTED

There is correlation between disease and constitution. That is why it is most important to study different constitution's influences on related diseases. The Yang deficiency constitution is linked to a series of cold symptoms characterized by a cold body and limbs owing to an insufficiency of Yang qi, which fails to warm the body and leads to a Yang deficiency-induced internal cold (cold-intolerant) [2]. The traits of Yang deficiency constitution and its diagnostic criteria proposed by Professor Wang Qi can be used as its diagnostic basis. Yang deficiency constitution is reflected in five aspects: (i) physical feature: flabby muscles; (ii) psychological feature: placid temper, introversion; (iii) common behavior: aversion to cold, cold hands and feet, preference for hot food, lassitude, pale enlarged tongue, and deep and slow pulse; (iv) ability to adapt oneself to external environment: having a preference for summer and dislike towards winter, susceptible to wind, cold, and dampness; (v) occurrence of disease: retention of phlegm fluid, swelling, and diarrhea, usually followed by cold transformation [3].

At present research on Yang deficiency constitution mostly focuses on genetics and metabolomics. The comparative results of the serum physiological and biochemical indices in balanced and Yang deficiency constitutions showed marked elevation of cAMP/cGMP, I B IL-IB, and thyroid stimulating hormone in Yang deficiency constitution, and significant reduction of adrenocorticotrophic hormone, cGMP, and FT4. This evidence illustrates functional reduction of the hypothalamus-pituitary-adrenal axis and hypothalamus-pituitary-thyroid axis in Yang deficiency constitution, which is related to the disturbed cyclic nucleotide system and immune dysfunction [4]. There is significant difference between balanced and Yang deficiency constitutions in peripheral blood gene expression detected by Professor Wang et al. The downregulation expression of thyroid hormone receptor beta (TRbeta) provides molecular biological interpretations for intolerance to cold in Yang deficiency constitution [5]. In summary, compared with balanced constitution, immunological surveillance is decreased in Yang deficiency constitution with upregulation expression of inflammatory cytokines and decreased genetic information transmission. Metabolomics study shows lactic acid, LDL, and fatty acid composition in Yang deficiency constitution is lower than that in balanced constitution. It means the energy metabolism level is lower in Yang deficiency constitution [6].

RETRACTED

However, there can be no definite conclusion about what particular systematic diseases will occur in Yang deficiency constitution. To explore the correlation between constitution and disease we try to do gene experiments by using mRNA profiling to find out the molecular biological ground in Yang deficiency constitution of young people, which is significant in constitution-disease study and prevention of disease.

## 2. Materials and Methods

### 2.1. Inclusion Criteria

(1) Chinese Han males and females, aged 18–28, were selected; (2) also selected were people who were able to meet the determinant standard for balanced constitution and Yang deficiency constitutions per the Chinese Medical Constitution 2008 Issued by the Chinese Association of TCM (frequent code: ZYYXH/T157-2009) (Table 1), with no clear-cut diagnosis of disease; and (3) informed consent was signed by the subjects.

Those who were not included had the following characteristics: (1) being not consistent with the above-stated inclusion guidelines or complicated with other types of constitution; (2) age < 18 years or > 28 years; (3) having severe heart, brain, liver, kidney disorders, or infectious disease and mental disorders; (4) being a carrier of virus or bacteria; (5) failing to sign the informed consent.

### 2.2. Subject Selection

The individuals were obtained at random from within the Beijing population. After identification of the constitution with the TCM theory and reexamination by TCM practitioners, those who met the inclusion guidelines were chosen. Among them 20% were reexamined by specialists to make sure of the veracity of constitution prediction.

After getting rid of the discrete samples, there were 28 subjects who were finally chosen for genetic variation analyzing, including 20 Yang deficiency constitution and 8 balanced constitution. The latter consisted of 2 males and 6 females, and the former 5 males and 15 females. There was no variation between the two groups in age (*P* = 0.395), sex (*χ*^2^ = 0.660, *P* = 0.5), and body mass index (*P* = 0.105) (Table 2).

### 2.3. Blood Samples and Experimental Procedures

The subjects had been informed of the objective, significance, and other related issues of the experiment and they agreed to sign the informed consent. The subjects were advised to abstain from alcohol consumption and to avoid fatigue in the 24-hour period immediately before the test. Female subjects were additionally advised not to test during menstruation. A 8 mL venous blood was collected before breakfast in the morning, and EDTA anticoagulation was performed. Leukocytes were separated by centrifugation at 3000 rgf for 5 min, and the peripheral blood mononuclear cells (PBMCs) were separated by gradient centrifugation for 2 hours. Then the isolated leukocytes were preserved in 1 mL Trizol reagent in a −80°C refrigerator. One week later the samples were delivered to the Bio Corporation (Beijing) to extract total RNA from the leukocytes. Using Affymetrix HG-U133Plus2.0 the gene expression profile of the peripheral blood was detected.

RETRACTED

### 2.4. Analysis of Microarray Data

The normalized ratio of gene expression signals was logarithmically transformed. Differentially expressed genes were identified by the linear models for microarray data (Limma) package in R software [7]. The cut-off criteria were set as follows: adjusted *P* value < 0.05 and gene expression fold change (FC) > 1.2 [8]. Hierarchical clustering was performed using average linkage method.

The Gene Ontology (GO) analysis was used to determine the biological function of the identified genes. The significance level of the functional GO terms was identified by Fisher's exact test (*P* < 0.05). The pathway enrichment analysis was used to confirm potential molecular interactions based on the KEGG database (http://www.kegg.jp/kegg/pathway.html) [9, 10]. The significance level of the enriched pathways was calculated using Fisher's exact test.

Gene functional annotations were generated using the canonical pathway module in Ingenuity Pathway (IPA) software (Ingenuity Systems; http://www.ingenuity.com/).

### 2.5. Statistical Analysis

The statistical analysis was carried out using the SPSS18 software. If the group comparison conformed to normal distribution, and the variance was uniform, the quantitative data were shown by mean *x* ± *s*. If it did not conform to the normal distribution, the rank sum test of the two dependent samples was done. The chi-square test was used for the enumeration data.

### 2.6. Ethical Review Committee Statement

The methods were carried out in accordance with the Declaration of the Helsinki Surgical Procedure. All experimental protocols were ethically approved by the Ethics Committee of Beijing University of Chinese Medicine Medical Research (Approval ID: 2012BZHYLL0301) and informed consent was obtained from all subjects.

## 3. Results

### 3.1. Gene Expression Profile Clustering Analysis

Yang deficiency constitution and balanced constitution can be classified in gene level (Figure 1). As all subjects were considered to be healthy, we collected* q* < 0.05 and fold change > 1.2 threshold for better analysis and found 909 upregulated and 1189 downregulated genes in Yang deficiency constitution. It indicated the gene expression profile clustering characteristics of these two constitutions were the same with the classification of TCM.

RETRACTED

### 3.2. Go Analysis

The GO analysis indicates the importance among the multifunction of the 43 remarkable GO expressions (*P* < 0.01); the most significant 4 GO categories for upregulated genes were response to nucleosome assembly, toll-like receptor 10 signaling pathway, toll-like receptor 5 signaling pathway, and stress-activated MAPK cascade (Figure 2). It is very visible that toll-like receptor disorder had significant and increased performance. In addition, the GO function also refers to the positive regulation of apoptotic process, innate immune response, and defense response to virus, which point to the apoptosis and immune response.

The GO function of downregulated genes was mainly about transcription, DNA-templated, regulation of transcription, DNA-templated, inflammatory response, and negative regulation of apoptotic process. Analysis of the GO Tree about the upregulated and downregulated path revealed the latter was in the majority and the immunoreaction was entirely downregulated (Figure 3). The GO Tree analysis indicated the 8 GO functions were related to the toll-like receptor's signal pathway (Figure 4). As a result, the DNA transfer ability downregulated glycerol metabolism and decreased inflammation, pressure, and so forth.

### 3.3. Ingenuity Pathway (IPA) Canonical Pathway Analysis

In Yang deficiency constitution there were 2098 differential genes in total. The significant 34 downregulated pathways were analyzed (*P* < 0.01). The downregulated differential gene pathways of Yang deficiency constitution after functional gathering presented mostly in signal transmission, for example, the TNF signaling pathway, NF-kappa B signaling pathway, FoxO signaling pathway, ErbB signaling pathway, MAPK signaling pathway, and the immune system pathway, for example, the NOD-like receptor signaling pathway, rheumatoid arthritis, toll-like receptor signaling pathway, inflammatory bowel disease (IBD), and intestinal immune network for IgA production (Figure 5).

When the differential genes gathered in 43 upregulated pathways (*P* < 0.05), there was incidence of immune disease, cancer, infectious disease, and endocrine dyscrasia. The immune problems included, for example, systemic lupus erythematosus, natural killer cell mediated cytotoxicity, Fc epsilon RI signaling pathway, and B cell receptor signaling pathway (Figure 6). Sometimes cancers were involved, for example, viral carcinogenesis, acute myeloid leukemia, chronic myeloid leukemia, colorectal cancer, and glioma. Infectious diseases included hepatitis B, influenza A, measles, legionellosis, and herpes simplex infection. It was different from the downregulated pathway gathering. The upregulated pathway of Yang deficiency constitution assembled at the endocrine system, for example, the prolactin signal pathway, female hormone signal pathway, and GnRH signal pathway.

RETRACTED

The maximal difference of downregulated pathway in comparison with the upregulated pathway was metabolism, which was chiefly related to glycometabolism, and so forth.

## 4. Discussion

The mRNA genomics of the population of Yang deficiency constitution aged from 18 to 28 were studied as well as the susceptible diseases. On the basis of the previous research by Yao Shilin, our sample size was expanded and focused on young people. We have found that Yang deficiency constitution often led to occurrence of immune diseases, such as enteritis due to immune problems, arthritis, lowered metabolism, and cancers. They all had genetic expression dysregulation molecular basis, which is of significance for research of “constitution-disease” correlation with Yang deficiency constitution and preventive treatment of disease.

The gene expression of Yang deficiency constitution indicated entirely lowered immunity. It has been found that, in comparison with balanced constitution, complete functional downregulation was seen in Yang deficiency constitution with maximal downregulated genes. The toll-like receptors mediated the negative regulation of inflammatory response signal pathway, which was activated by pathogens and quickly resulted in inflammatory response. It served to regulate innate and acquired immunoreaction. As you see Yang deficiency constitution is characterized by lowered immunity, but it also has higher immunoreaction and susceptibility to immune problems. Some researchers have proved hypofunction is seen in Yang deficiency constitution. For example, Qiyang et al. have found Lewis mouse kidney-deficiency constitution and its HPA function's imbalance [11]. The index of liver, kidney, and adrenal gland remarkably reduced (*P* < 0.01) as well as ACTH, CRH, c GMP, and Cort, 17OHCS (*P* < 0.01). Qi deficiency and Yang deficiency constitutions are the risk factors of chronic fatigue syndrome [12].

The downregulated differential genes mainly gathered at the disturbed pathways of the immune and metabolic systems. Immune disorders such as rheumatoid arthritis, inflammatory bowel disease (IBD), and intestinal immune network for IgA production occurred. It conforms to the fact that arthritis due to cold and dampness and diarrhea usually occur in people with Yang deficiency constitution. Some research showed that ulcerative colitis with the kidney Yang deficiency syndrome could be characterized by the reduction of serum Treg and TGF-beta 1 levels, which represented a depression of immune tolerance. About Yang deficiency constitution and arthritis Jing Pingfu found Yang deficiency constitution was the risk factor of knee osteoarthritis, which induced Sox9 and lowered expression of Co12al [13]. Insufficient Yang qi and insecurity of defensive Yang fail to warm the muscles against invasion by external wind, cold, and dampness, leading to impediment like arthritis caused by qi and blood blockage in meridians in people with Yang deficiency constitution.

RETRACTED

Lowered metabolism is an important manifestation of mRNA expression in Yang deficiency constitution, which involves mainly carbohydrate metabolism, glycan synthesis, and lowered metabolism. The elated genes are MTMR2, FBP1, C12orf5, PFKFB3, TPI1, ALDOC, HS2ST1, XYLT1, B3GAT2, B3GALT6, HS3ST3B1, and CSGALNACT2. This is a molecular evidence of intolerance to cold in Yang deficiency constitution. At the same time, it predicts Yang deficiency constitution is susceptible to hypoglycemia. In addition, nuclear magnetic resonance- (NMR-) based metabolomics were applied to study Yang deficiency constitution by analyzing metabolic profiling of the serum and urine. Compared with the balanced constitution, the contents of lactate (FA) and unsaturated fatty acid (UFA) are lower while the contents of glutamine, glucose, phosphatidylcholine (PtdCho), and high density lipoprotein (HDL) are higher in serum of Yang deficiency constitution, and the content of creatinine is lower while the contents of lactate, DMA, citrate, and hippurate are higher in the urine of Yang deficiency constitution. Yang deficiency constitution has some metabolism disorders of energy, lipid, and glucose and also has organic functional changes, which further reveals disturbed glucose and lipid metabolism [14]. In another report, deregulated genes in the Yang deficiency constitution were found to be enriched for energy, lipid, and glucose metabolism and changes of organ functions.

Yang deficiency constitution is also the risk factor of cancer caused by dysfunction of the zang-fu organs and decreased immune function. It is a debilitated condition, easy to contract cancers compared to people with balanced constitution. Traditional Chinese medicine believes incidence and progress of cancer is closely related to diminish healthy qi and too strong pathogenic factors. Researches done by Sili et al. showed that the related genes of aged kidney-deficiency constitution came down with ageing and occurrence of cancer and reproductive diseases, which illustrates the relationship between kidney-yang deficiency and brain-kidney relationship. In addition, aged women usually suffered from diminished meridian qi [15]. Alongside the increase of age of breast cancer females with Yang deficiency constitution, their meridian qi is much lower [16]. Older women have lower meridian qi. The more severe the symptoms are, the lower the overall meridian qi is. The researches also showed the estrogen and prolactin pathways were upregulated. According to experiments, by means of increasing NIS gene expression prolactin, estrogen, cAMP, and stimulants retinoic acid and glucocorticoid enhanced iodine uptake of the breast cancer cells [17].

RETRACTED

Researches by Moore et al. indicated markedly higher total estrogen/estrogen metabolite concentrations in postmenopausal US women (Asian Americans) than in Shanghai women may partly explain higher breast cancer rates in the United States [18]. Estrogen can regulate the functions of nearly all immunocyte subsets, which may contribute to the development of autoimmune thyroid diseases and thyroid cancer. ERalpha activation seems to exacerbate the development of thyroid cancer, while wild-type ERbeta (ERbeta1) plays a protective role against thyroid cancer [19]. These results suggest that estrogen may play a role in androgen-independent prostate cancer cell proliferation through a novel pathway, involving ERbeta-mediated activation of beta-catenin [20]. Furthermore, the Yang deficiency constitution exhibits decreased levels of mRNA expression for several key nuclear receptor coactivators including steroid receptor coactivator I (SRC1), steroid receptor coactivator 3 (SRC3), cAMP-response element-binding protein (CREB), and binding protein (CBP), and mediator is significantly decreased [5].

Since the above study involves the healthy population, it is necessary to experience a long-term observation to confirm the significance of earlier reminder. Our study of Yang deficiency constitution frequently tells us there exists lowered immunity in them. But each time there is differential molecular expression, which may be related to sample number and age.

## 5. Conclusions

Based on our genome researches, we have further analyzed the correlated disease risk of Yang deficiency constitution, that is, immune problems, cancer, arthritis, enteritis, and lowered metabolism, which conforms to clinical manifestations in Yang deficiency constitution. The present study concerns Yang deficiency constitution under absence of disease, which proves existence of Yang deficiency constitution and lays molecular foundation for study of “constitution-disease.”

However, the genetic basis, physiological features, and clinical significance of this variation were largely undefined. In comparison, the TCM constitution system provides a conceptual framework and rich resources to study the classification of healthy individuals and related disease risks.

RETRACTED

## Figures and Tables

**Figure 1:** Clustering analysis of differentially expressed genes between Yang deficiency and balanced constitutions. Clustering analysis was performed using a hierarchical, average linkage algorithm. Red and green colors represent upregulation and downregulation, respectively.

**Figure 2:** The most significant enriched GO cluster of upregulated genes in Yang deficiency constitution compared to balanced constitution.

**Figure 3:** The most significant enriched GO cluster of downregulated genes in Yang deficiency constitution compared to balanced constitution.

**Figure 4:** Go Tree. The significant enriched GO cluster of up- and downregulated genes in Yang deficiency constitution compared to balanced constitution. The red color indicates the upregulated function while the green color the downregulated function. The yellow color shows the differential genes, either upregulated or downregulated ones.

**Figure 5:** IPA canonical pathway analysis. The significant enriched pathway cluster of downregulated genes in Yang deficiency constitution compared to balanced constitution.

**Figure 6:** IPA canonical pathway analysis. The significant enriched pathway cluster of upregulated genes In Yang deficiency constitution compared to balanced constitution.

**Table 1:** Diagnostic standards for Yang deficiency and balanced Constitutions.

	Yang deficient constitution	Balanced constitution
Main characteristics	Cold intolerance	Energetic
	Cold hands, feet,	Without all symptoms or characteristics of above constitutions
	stomach, and waist	
	Prefer hot food and drinks	
	Susceptible to cold	
Secondary characteristics	Watery stool	Good sleep
	Fat	Cold tolerance
	Whitish skin	Good memory
	Nocturia	
	Tender and pale tongue	

**Table 2:** The baseline information.

Group	Gender^*∗*^		Age	Body mass index
	Male	Female		
A (balanced constitution)	2	6	23.50 ± 2.50	24.214 ± 4.186
B (Yang deficiency constitution)	5	15	23.50 ± 5.50	21.042 ± 4.175
*χ*^2^	0.660			
*t*-test	0.5		0.395	0.105
